The article "Targeted Perioperative Nursing Combined with Propofol and Fentanyl for Gynecological Laparoscopic Surgery" was retracted in 2023. Reasons: unreliable results or conclusions; lack of ethics approval or compliance; concerns about the data; concerns about the peer review.

# Targeted Perioperative Nursing Combined with Propofol and Fentanyl for Gynecological Laparoscopic Surgery

**DOI:** 10.1155/2022/1257260

**Published:** 2022-10-15

**Authors:** Xue-Yu Yun, Shu-Juan Chen, Qiu-Wu Zheng

**Affiliations:** ^1^Operation Room, The Second Affiliated Hospital of Hainan Medical College, Haikou 570216, China; ^2^Operation Room, Hainan Modern Women and Children's Hospital, Haikou 570206, China

## Abstract

**Objective:**

The aim of this study is to investigate the clinical effects of targeted perioperative nursing combined with propofol and fentanyl in gynecological laparoscopic surgery.

**Methods:**

Patients who were admitted to our hospital for gynecological laparoscopic surgeries from October 1, 2019 to November 30, 2021 were included in this retrospective study. Patients in group A received routine propofol and fentanyl. Patients in group B received targeted perioperative nursing on the basis of interventions in group A. The anesthetic effects, clinical indicators, mental health status, and adverse reactions were compared between the two groups.

**Results:**

A total of 84 qualified patients were retrieved. The total effective anesthesia rate, extubation time, operation time, consciousness recovery time, intraoperative blood loss, hospital stay, SAS score, SDS score, health status indicators, and adverse events in group B were all significantly better than those in group A (*P* < 0.05 for all comparisons).

**Conclusion:**

Combined intervention (propofol + fentanyl + targeted perioperative care) for gynecological laparoscopic surgery patients has a significant anesthesia effect, which can effectively improve the patient's clinical indicators and mental health status and can also reduce the occurrence of adverse events. It has good safety and can be widely used in clinical practice.

## 1. Introduction

With the continuous development of clinical minimally invasive and endoscopic techniques, laparoscopic surgery has been widely used in the gynecological field due to its advantages of fewer traumas, less pain, and faster recovery from surgery [1]. The advantages of propofol and fentanyl, such as the rapid onset of anesthesia and no accumulation of anesthetic effect, make them widely used in gynecological laparoscopic surgeries [2, 3]. The fast development of laparoscopic surgery also leads to higher requirements for nursing staff in clinical practice, so as to improve the quality of nursing services and promote a more harmonious relationship between doctors and patients, which is beneficial to postsurgical recovery to a certain extent [4, 5].

Anxiety and depression are commonly seen in postsurgical and cancer patients, especially in the elderly and females [6, 7]. Therefore, in this study, we retrieved patients who were admitted to our hospital and received gynecological laparoscopic surgeries and further analyzed the clinical effects and mental status after the combined postsurgical intervention (propofol + fentanyl + targeted perioperative care), aiming to provide a basis for clinical care plan in patients after gynecological laparoscopic surgeries.

The article "Targeted Perioperative Nursing Combined with Propofol and Fentanyl for Gynecological Laparoscopic Surgery" was retracted in 2023. Reasons: unreliable results or conclusions; lack of ethics approval or compliance; concerns about the data; concerns about the peer review.

## 2. Materials and Methods

Patients who received gynecological laparoscopic surgeries at our hospital from October 1, 2019 to November 30, 2021 were retrieved and divided into group A and group B. Patients in group A received routine surgical intervention, while patients in group B were given targeted perioperative care on the basis of intervention in group A. Inclusion criteria [8]: (1) all included patients met the corresponding criteria for gynecological laparoscopic surgery; (2) aged between 18 and 80 years old; (3) the clinical data of all included patients were complete. (4) Signed the informed consent form. Exclusion criteria [9]: (1) patients with severe mental disorders or clouded consciousness; (2) patients with respiratory diseases; (3) patients with certain contraindications or allergic history to anesthetics. This study was approved by the Ethics Committee of our hospital

Anesthesia intervention: The patient was first given in of atropine 0.5 mg before surgery. Secondly, the clinical signs of the patient were monitored immediately after entering the operating room, and 0.04 mg/kg midazolam, 2 mg/kg propofol and, and 0.4 ug/kg fentanyl were used to induce anesthesia, and then tracheal intubation was performed to assist ventilation. Finally, anesthesia was maintained with 0.5 ug/kg/min fentanyl and 4 mg/kg/h propofol, which was terminated 30 min before the completion of surgery.

Patients in group A received routine surgical intervention, while patients in group B received targeted perioperative nursing on the basis of the intervention in group A [10]. The specific steps were: (1) Preoperative intervention: patients were prone to anxiety and depression and other adverse psychological emotions before surgery. Therefore, nursing staff should actively communicate with patients at this time and enhance their confidence in treatment by patiently informing patients of successful anesthesia cases. At the same time, nursing staff should also make sufficient preparations for surgery and prepare ECG monitors, ventilators, and all necessary surgical instruments before surgery. (2) Intervention during operation: after the patient enters the operating room, the nursing staff should provide psychological intervention with the patient in time to relieve their negative psychological emotions. A series of unexpected situations may occur during the operation, so the nursing staff should focus on monitoring the patient's physical indicators. At the same time, it is also necessary to timely solve the problems of aspiration and reflux that might occur during the operation. (3) Postoperative intervention: after the operation, the nursing staff should reassure the patient's psychological state, instruct the patients to remain in a supine position after returning to the ward, and pay close attention to their vital signs until they return to normal. At the same time, it is necessary to avoid slippage of the drainage tube and record the status, color, smell, and drainage volume of the drainage material in detail.

The article "Targeted Perioperative Nursing Combined with Propofol and Fentanyl for Gynecological Laparoscopic Surgery" was retracted in 2023. Reasons: unreliable results or conclusions; lack of ethics approval or compliance; concerns about the data; concerns about the peer review.

### 2.1. Evaluation of Anesthesia Effect

Significant effect: the patient's anesthesia induction state is stable, the depth of anesthesia maintenance is reasonable, and the state is stable during recovery; normal effect: the patient's anesthesia induction state is relatively stable, the depth of anesthesia maintenance is reasonable, and mild agitation occurs during recovery; terrible effect: the patient's anesthesia induction state unstable, unreasonable depth of anesthesia maintenance, severe agitation during recovery. Total effective effective anesthetic rate = (Significant + Normal)/total number of cases × 100% [11, 12].

### 2.2. Evaluation of Clinical Indicators

The extubation time, operation time, consciousness recovery time, intraoperative blood loss, hospitalization days, and adverse events of the two groups of patients were recorded and compared [13].

### 2.3. Assessment of Mental Health Status

The anxiety and depression status of the patients were assessed by the Self-rating Anxiety Scale (SAS) and Self-Rating Depression Scale (SDS) scores, respectively. A SAS score ≥50 indicated that the patient had anxiety, and a SDS score ≥53 points indicates that the patient had depression [14, 15].

### 2.4. Statistical Methods

Data were analyzed by SPSS21.0 (IBM, Armonk, USA). The enumeration data were represented by *n*(%) and analyzed by *χ*^2^ test, and the measurement data were expressed by mean ± SD and analyzed by *t*-test, and the difference was determined as significant if a 2-sided *P* < 0.05.

## 3. Results

A total of 84 qualified patients were retrieved. The average age was (35.94 ± 5.56) years in group A (*n* = 42), and (36.14 ± 4.82) years in group B (*n* = 42). The clinical characteristics of the enrolled patients were detailed in Table 1, which showed no significant differences in age, weight, or primary disease composition between the two groups (*P* > 0.05).

The article "Targeted Perioperative Nursing Combined with Propofol and Fentanyl for Gynecological Laparoscopic Surgery" was retracted in 2023. Reasons: unreliable results or conclusions; lack of ethics approval or compliance; concerns about the data; concerns about the peer review.

### 3.1. Comparison of Anesthesia Effects

The total effective anesthetic rate of group B after this combined intervention was 88.12% (37/42), which was more significant than that of group A (73.81%, 31/42) (*P* < 0.01, Table 2).

### 3.2. Comparison of Clinical Indicators

There were significant differences in the extubation time (7.12 ± 2.32 min vs 5.32 ± 1.56 min), operation time (76.33 ± 11.39 min vs 100.76 ± 22.67 min), consciousness recovery time (10.32 ± 2.25 min vs 5.78 ± 1.64 min), intraoperative blood loss (98.53 ± 37.48 ml vs 115.51 ± 28.54 ml), hospital stay (7.45 ± 2.32 days vs 5.64 ± 1.64 days) between group A and group B (*P* < 0.01). Details are shown in Table 3.

### 3.3. Comparison of Mental Health Status

At admission, there were no significant differences in SAS score (70.38 ± 6.67 vs 71.21 ± 7.83) or SDS score (75.12 ± 7.56 vs 74.78 ± 8.34) between group A and group B. After intervention, there were significant differences in the SAS score (55.34 ± 3.45 vs 48.44 ± 3.12, *P* < 0.05) and SDS score (61.34 ± 5.41 vs 50.41 ± 3.26, *P* < 0.01) between group A and group B. See Table 4 for details.

### 3.4. Comparison of Adverse Events

There were no severe adverse symptoms in the two groups of patients after interventions, which indicated the safety of the intervention program. The total incidence of adverse events in group B was 9.52% (6/42), which was significantly lower than that of group A (28.57%, 12/42) (*P* < 0.01). See Table 5 for details.

## 4. Discussion

Laparoscopic surgery is a common minimally invasive surgery in clinical practice, and it has received widespread attention and recognition due to its small postoperative trauma, fewer complications, and faster recovery [16, 17]. Clinically, propofol and fentanyl are used to anesthetize patients with good effect. While propofol has a fast onset and strong controllability, and will not cause much impact on hemodynamics, fentanyl has a good analgesic effect [18, 19]. The application of targeted perioperative care in the perioperative period of surgical patients can improve the patient's compliance and complete the operation more smoothly [16, 20]. In this study, we found that the total effective anesthesia rate, extubation time, operation time, consciousness recovery time, intraoperative blood loss, hospital stay, SAS score, SDS score, health status indicators, and adverse events in group B were all significantly better than those in group A. This shows that propofol + fentanyl + targeted perioperative care is superior to routine surgical intervention.

Patients undergoing gynecological laparoscopic surgery usually have different degrees of negative psychological emotions, mainly because of the uncertainty of the implementation of the operation, which leads to a series of concerns and worries about the disease prognosis and recovery process. Patients are afraid of surgery, so effective psychological intervention is of great significance to relieve the patient's negative emotions [21, 22]. In this study, there were no significant differences in SAS score or SDS score between the two groups at admission, but there were significant differences in SAS score or SDS score after intervention, which shows that the intervention program of group B can greatly improve the patient's mental health and speed up the recovery. The application of targeted perioperative care might be promising in more severe cases, such as brain injury, fulminant hepatitis, infection, and so on [23–30].

The article "Targeted Perioperative Nursing Combined with Propofol and Fentanyl for Gynecological Laparoscopic Surgery" was retracted in 2023. Reasons: unreliable results or conclusions; lack of ethics approval or compliance; concerns about the data; concerns about the peer review.

All in all, the combined intervention (propofol + fentanyl + targeted perioperative care) for gynecological laparoscopic surgery patients has a significant anesthetic effect, which can effectively improve the patient's clinical indicators and mental health status and reduce the occurrence of adverse reactions. It has good safety and can be widely used in clinical practice.

## Figures and Tables

**Table 1:** Comparison of the clinical characteristics.

Group	Case	Age (years-old)	Weight (kg)	Primary disease (case)		
				Uterine fibroids	Ectopic pregnancy	Ovarian cyst
A group	42	35.94 ± 5.56	51.3 ± 1.85	8	13	21
B group	42	36.14 ± 4.82	50.4 ± 2.17	10	12	20
*χ * ^2^ * /t/u*		0.453	0.335		0.331	
*P*		0.521	0.572		0.632	

**Table 2:** Comparison of anesthesia effect [*n* (%)].

Group	Significant;	Normal	Terrible	Total effective rate
A group (*n* = 42)	18 (42.86)	13 (30.95)	11 (26.19)	31 (73.81)
B group (*n* = 42)	23 (54.76)	14 (33.33)	5 (11.91)	37 (88.12)
*χ * ^2^		—		6.985
*P*		—		<0.01

**Table 3:** Comparison of clinical indicators (days, mean ± SD).

Project	A group (*n* = 42)	B group (*n* = 42)	*t*	*P*
Duration of extubation (min)	7.12 ± 2.32	5.32 ± 1.56	10.764	<0.01
Operation time (min)	76.33 ± 11.39	100.76 ± 22.67	15.564	<0.01
Consciousness recovery time (min)	10.32 ± 2.25	5.78 ± 1.64	9.431	<0.01
Intraoperative blood loss (ml)	115.51 ± 28.54	98.53 ± 37.48	18.445	<0.01
Hospital days (d)	7.45 ± 2.32	5.64 ± 1.78	4.112	<0.01

**Table 4:** Comparison of mental health status of two groups of patients before and after intervention (mean ± SD).

Group	A group (*n* = 42)	B group (*n* = 42)	*t*	*P*
*SAS score*				
On admission	70.38 ± 6.67	71.21 ± 7.83	0.564	>0.05
After intervention	55.34 ± 3.45	48.44 ± 3.12	5.564	<0.01

*SDS score*				
On admission	75.12 ± 7.56	74.78 ± 8.34	0.575	>0.05
After intervention	61.34 ± 5.41	50.41 ± 3.26	7.563	<0.01

**Table 5:** Comparison of the occurrence of adverse events [*n* (%)].

Group	Shortness of breath	Nausea and dizziness	Mania	Total incidence
A group (*n* = 42)	3 (7.14)	3 (7.14)	6 (14.28)	12 (28.57)
B Group (*n* = 42)	1 (2.38)	1 (2.38)	2 (4.76)	6 (9.52)
*χ * ^2^		—		4.657
*P*		—		<0.01

The article "Targeted Perioperative Nursing Combined with Propofol and Fentanyl for Gynecological Laparoscopic Surgery" was retracted in 2023. Reasons: unreliable results or conclusions; lack of ethics approval or compliance; concerns about the data; concerns about the peer review.

## Data Availability

The data used to support the findings of this study are available from the corresponding author upon request.
